# Antitumor Effects of 10058-F4 and Curcumin in Combination Therapy for Pancreatic Cancer In Vitro and In Vivo

**DOI:** 10.1155/2022/1620802

**Published:** 2022-03-24

**Authors:** Zhang Jie, Zhang Jinna, Zhang Jingjun, Li Pengcheng, Yang Fang, Chen Qinyang, Chen Taiyu, Jiang Hequn, Ren Tao

**Affiliations:** ^1^Clinical Medical College and The First Affiliated Hospital of Chengdu Medical College, Si Chuan, China; ^2^No.4 West China Teaching Hospital of Si Chuan University, Si Chuan, China; ^3^The People's Hospital of JianYang City, Si Chuan, China; ^4^Chengdu Medical College, Si Chuan, China; ^5^South China Hospital of Shenzhen University, Guang Dong, China

## Abstract

**Background:**

Pancreatic cancer (PC) stands out as one of the most lethal cancers. Due to late diagnosis, only a fraction of patients can be resected. Although it still has significant adverse effects and poor results, the treatment is connected with better overall survival than the prior treatment. Thus, new alternative therapy for advanced PC is needed. *Materials/Methods*. The impact of 10058-F4 and curcumin combination therapy on apoptosis and cell growth in SW1990 pancreatic cancer cells were determined in vitro using the CCK-8 assay and flow cytometry of Annexin V-FITC/PI, and the in vivo antitumor effect was determined utilizing SW1990-bearing pancreatic tumor mouse models induced by subcutaneous implantation.

**Results:**

At concentrations of (10 mol/L+2 mol/L), 10058-F4+curcumin obtained the highest rate of SW1990 cell death, and they had a beneficial effect on SW1990 pancreatic tumor-bearing animals. Furthermore, c-Myc, Akt phosphorylation, and the expression of apoptosis-related molecular were reduced, and the combination therapy modified the expression of apoptosis-related molecular.

**Conclusions:**

In vitro and in vivo, the combination of 10058-F4 plus curcumin has antipancreatic cancer actions that are substantially effective.

## 1. Introduction

Pancreatic ductal adenocarcinoma (PDAC), having a 5-year survival rate of only 9%, is one of the fatal human cancers [1]. The only treatment that can potentially offer a cure for pancreatic cancer is surgical resection [2]. Immune checkpoint blockade therapies that are beneficial in other cancers have failed to benefit randomly selected PDAC populations in phase III trials [3]. As a proto-oncogene, c-Myc has been found to be activated in a variety of animal and human malignancies and is required for the metabolism, differentiation, apoptosis, and cell proliferation [4]. Previous research has established that overexpression of c-Myc has an involvement in the development and progression of PDAC [5, 6]. c-Myc downregulation impedes the development of PDAC [7, 8].

A small-molecule inhibitor of c-Myc-Max dimerization, referred to as 10058-F4, has been demonstrated to reduce cellular proliferation, increase apoptosis, and induce chemosensitivity [9–11]. Furthermore, no substantial tumor growth inhibition was observed after intravenous injection of either 20 or 30 mg/kg 10058-F4 into mice. The quick metabolism and low tumor concentration of 10058-F4 may have resulted in its lack of considerable antitumor effect in tumor-bearing mice [12]. The anticancer action of 10058-F4 has been reported in PDAC cell lines, and 10058-F4 therapy sensitizes PANC-1 and SW1990 cells to gemcitabine. In a subcutaneous xenograft model, 10058-F4 did not affect pancreatic carcinogenesis; however, when paired with 10058-F4, the anticancer impact of gemcitabine is more substantial [13].

Curcumin is a pure crystalline yellow pigment derived from the turmeric plant [14]. Curcumin possesses antitumor, antiangiogenesis, antiproliferative, and anti-inflammatory activities without causing cytotoxicity in normal cells [15, 16]. Curcumin has the potential to cause apoptosis in cancer cells [17]. Apoptotic proteins, inflammatory cytokines, transcription factors, and growth factors have all been shown to be modulated by curcumin. It can be an effective cancer therapy agent when used alone or in combination with other drugs [18]. Two reports indicate that curcumin regulates c-Myc [19, 20]. Curcumin inhibits gastric cancer cell proliferation by inhibiting the c-Myc/H19 pathway [19]. It can also have a strong inhibitory effect in three prostate cancer cell lines by upregulating miR-34a and downregulating *β*-catenin and c-Myc levels [20]. Curcumin has been found to have anticancer properties in PDAC cell lines. Interacting with the miR-340/XIAP signaling pathway has been demonstrated to promote apoptosis in pancreatic cancer cells in vitro [21].

Curcumin can also block EGF-induced pancreatic cancer cell invasion and migration by inhibiting the EGF/EGFR signaling pathway and downstream signaling molecules, for instance, ERK and Akt [22]. Curcumin inhibits the PI3K/Akt/NF-*κ*B signaling pathway, preventing SOD-driven H_2_O_2_-induced pancreatic cancer metastasis [23]. Curcumin is shown to sensitize gemcitabine-resistant PDAC cell lines via an inhibitory effect on the PRC2-PVT1-c-Myc axis [24]. Such studies suggest that using curcumin in combination with chemotherapy to overcome chemoresistance in PDAC has therapeutic efficacy. Curcumin may inhibit c-Myc and improve the clinical therapeutic potential of the c-Myc inhibitor 10058-F4 in pancreatic cancer cells. This study used curcumin or 10058-F4 alone or in combination to treat SW1990 cells in vitro and in vivo. Curcumin therapy sensitized SW1990 cells to 10058-F4 for the first time.

## 2. Materials and Methods

### 2.1. Chemicals and Cell Culture

The Chinese Academy of Sciences (CAS) Cell Bank provided the pancreatic cancer cell lines PANC-1, SW1990, BxPC3, Capan-1, and Capan-2 (Shanghai, China). In a 5% CO_2_ cell culture incubator at 37°C, cells were grown in high-glucose DMEMR or PMI-1640 media supplemented with 10% fetal bovine serum (FBS; Gibco) and 1% penicillin or streptomycin. In dimethylsulfoxide (DMSO) (Sigma), 100 mM stock solutions of curcumin and 100 mM stock solutions of 10058-F4 (Selleck) were produced.

### 2.2. Cell Proliferation Assay

5,000 SW1990 cells were planted in individual wells of a 96-well plate, in 100 *μ*l completed DMEM medium. Cells were monotreated with either 10058-F4 (10 *μ*M) or curcumin (5 *μ*M) for 48 hours before cotreatment with both 10058-F4 and curcumin. The Cell Counting Kit-8 (CCK-8, Dojindo) was employed to analyze cell proliferation, following the protocol elaborated by the manufacturer. Each well was filled with 10 *μ*l CCK-8 solution and 90 *μ*l DMEM. After oscillating for 15 seconds, the cell absorbance was measured at a wavelength of 450 nm (OD450) 2 hours later.

### 2.3. Colony Formation Assay

Different groups of people took part in the colony formation test. SW1990 cells were trypsinized and grown in 6-well plates at a density of 1,000 cells per well. Four groups of cells were created. The cells were monotreated with 10058-F4 (10 *μ*M) or curcumin (5 *μ*M) for 24 or 72 hours, later cotreated with 10058-F4 and curcumin twice. After 2 weeks, the colonies were fixed for 15 minutes with 4% (*w/v*) formaldehyde and stained for 15 minutes with 0.1% (*w/v*) crystal violet. Chemiluminescent image analysis photographs the colonies (Bio-Rad, ChemiDoc Touch, USA).

### 2.4. Flow Cytometry

SW1990 cells were trypsinized and grown in 6-well plates at a density of 2 × 10^5^ cells per well. The cells were separated into four groups and treated with either 10058-F4 (10 *μ*M) or curcumin (5 *μ*M) alone or in combination for 48 hours. Trypsinization was used to harvest cells from four groups, and the cell density was maintained at 5 × 10^5^ cells per ml. Centrifugation at 1200 rpm was used to wash the cell samples with phosphate-buffered saline (PBS). Following that, the Annexin V-FITC/PI Apoptosis Detection Kit (BD Pharmingen, CA, USA) was used to stain the cell samples as mentioned in the instructions provided by the manufacturer. After 30 minutes at 37°C in the dark, the stained cells were counted by making use of a FACS Calibur (BD Biosciences, San Jose, CA, USA) and analyzed through FlowJo software v.7.6.5 (Tree Star, OR, USA).

### 2.5. Xenograft Models of SW1990 Cells in Nude Mice

12 male BALB/c nu/nu mice (5 weeks old and weighing around 18–22 g) were acquired from Shanghai Beijing Vital River Laboratory Animal Technology and kept within 12/12 h light/dark cycles with unrestricted supply of water and rat chow. The Medical Experimental Animal Care Commission approved the experimental methodology of Chengdu Medical College's First Affiliated Hospital. For producing the subcutaneous tumors, SW1990 cells (1 × 10^7^ cells) in 0.2 ml PBS were injected into the right flank of test mice. Following one week, the mice were divided into four groups: the control group (with intraperitoneal and intravenous injections of equivalent solvent), the 10058-F4 group (with intravenous injections of 20 mg/kg 10058-F4 every other day), the curcumin group (with intraperitoneal injections of 25 mg/kg curcumin every other day), and the combination group (with intravenous injections of 20 mg/kg 10058-F4 and 25 mg/kg curcumin. Curcumin (25 mg/kg) was dissolved in 80% ddH_2_O, 10% PEG300, 5% Tween 80, and 5% DMSO following the manufacturer's protocol. Dissolution of 10058-F4 (20 mg/kg) in a mixture of ethanol, Cremophor EL, and saline (1 : 1:8 v/v/v) to a final concentration of 2 mg/ml yielded the dosing solutions. Three mice from each group were slain three weeks later to obtain the implanted tumors.

#### 2.5.1. Immunohistochemistry and Terminal Deoxynucleotidyl Transferase d-UTP Nick End Labeling (TUNEL) Staining

To eliminate endogenous peroxidase activity, the xenograft tumor tissues were cut into 4 *μ*m thick slides after being embedded in paraffin and then treated with xylene to remove paraffin and rehydrate. The slides were incubated for 30 minutes at room temperature with 5% goat serum. A rabbit anti-PCNA antibody was used to treat the slides after being washed (1 : 100, Abcam, Cambridge, UK). As a final step, the Thermo Fisher Scientific HRP DAB (UltraVision Quanto Detection System) was employed for the detection of PCNA expression. Mayer's hematoxylin (Sigma-Aldrich, St. Louis, MO) was employed for counterstaining the slides, and neutral resins (Thermo Fisher Scientific, Pittsburgh, PA, USA) were used to attach coverslips. This study used the TdT-mediated d-UTP labeling approach to assess TUNEL staining, which was conducted in accordance with the manufacturer's instructions (Roche, Applied Biosystems). Apoptotic cell DNA fragments were tagged at free 3′-OH DNA ends and strand breaks, respectively. An antifluorescein antibody coupled with alkaline phosphatase was used to detect fluorescein. Light microscopy was used to examine the stained cells after the reaction with the substrate had taken place.

### 2.6. Western Blot

Using RIPA lysis buffer and protease/phosphatase inhibitor cocktail (MedChemExpress, NJ, USA) with 1 mM phenylmethyl sulphonyl fluoride PMSF (Beyotime Biotech, Shanghai, China), the whole protein in each cell sample was extracted and quantified with a BCA protein assay (Beyotime Biotech, Shanghai, China). After blocking the protein with the primary antibodies against c-Myc, SOX2, p-Akt (Ser473), Akt, MCL-1, Bcl-2, FAS, and cleaved-caspase 3 beta-actin (1 : 1000, Cell Signaling Technology, Danvers, MA USA), the incubation period was extended overnight at 4°C. Secondary antibody conjugated to HRP (Beyotime Biotech, Shanghai, China, 1 : 4000) was incubated for 2 hours at room temperature with protein. The eECL Western blot kit (Beyotime Biotech, Shanghai, China) was utilized to detect the protein.

## 3. Results

### 3.1. High Expression of c-Myc in Pancreatic Cancer

In prior research, the c-Myc gene is substantially expressed in pancreatic cancer cells [7, 8, 13]. It was shown that human pancreatic cancer cells overexpress c-Myc, as were normal pancreatic epithelial cell hTERT-HPNE in our investigation of 5 human pancreatic cancer cell lines (PANC-1, SW1990, BxPC3, Capan-1, and Capan-2 cells), as shown in Figure 1(a).

### 3.2. Curcumin Sensitized the Anticancer Influence of 10058-F4 in Pancreatic Cancer Cells

10058-F4 is a c-Myc inhibitor [9, 10]. Curcumin also inhibits c-Myc [19, 20]. To further confirm the therapeutic value of targeting c-Myc, we attempted to sensitize the anticancer influence of 10058-F4 using curcumin and investigated the degree of inhibition of c-Myc using 10058-F4, curcumin, or a combination of both. First, we checked cell viability in 10058-F4 curcumin and combined treating SW1990 cells by detecting OD450 with CCK-8 reagent. Cell viability was gradually inhibited in the combination group (Figure 1(b)). The clonogenic assay results also confirmed the potent anticancer effect of the combination (Figure 2(a)). Since 10058-F4 and curcumin can induce apoptosis [9, 17], we postulated that the combination of 10058-F4 and curcumin might induce server apoptotic death in SW1990 cells. We used flow cytometry to directly examine the effects of 10058-F4 or curcumin treatment on early (Annexin V+/PI-) and late (Annexin V+/PI+) apoptosis on SW1990 cells. According to our findings, curcumin improved the sensitivity of 10058-F4 to SW1990 cells (Figure 2(b)).

### 3.3. In Vivo, Curcumin Increased the Therapeutic Efficacy of 10058-F4 in Pancreatic Cancer Cells

To further explore the effect of cotreatment with curcumin and 10058-F4 in vivo, SW1990 cells were implanted subcutaneously in Balb/c nu/nu mice (*n* = 3 for each group); one week later, the mice were treated with 10058-F4 by vein injection or curcumin alone by intraperitoneal injection or both 10058-F4 and curcumin every 3 days. After continuously treating the indicated drugs for 3 weeks, the combined group's average tumor weight was significantly lighter than in the monotherapy groups (Figure 3).

Additionally, PCNA and TUNEL labeling were used to detect cells in growth or death, respectively. Compared to the control group, the 10058-F4 and curcumin-treated groups have reduced the number of PCNA-positive cells and increased TUNEL-positive cells, but not the 10058-F4-treated group (Figure 4). As a result, our data established that the combination of 10058-F4 and curcumin had significant anticancer activity in vivo.

### 3.4. Curcumin Increased the Susceptibility of Pancreatic Cancer Cells to 10058-F4 by Inhibiting the Akt-Mediated Apoptotic Pathway

Accumulating evidence has shown that the Akt expression and phosphorylation are reduced by curcumin [22, 23] and upregulated by c-Myc [25]; we evaluated the expression levels of c-Myc, p-Akt, and Akt. As a result, we examined the expression levels of the apoptosis-related proteins Mcl-1, Bcl-2, Fas, and cleaved-caspase 3. Our findings showed that c-Myc and Akt phosphorylated protein levels were lower in SW1990 cells undergoing treatment with a combination of medicines than in cells treated with 10058-F4 alone (Figure 5(a)). Furthermore, the protein levels of Mcl-1 and Bcl-2 were dramatically reduced, whereas Fas and cleaved-caspase 3 were significantly enhanced in the combo treatment group (Figure 5(b)).

## 4. Discussion

The oncogene c-Myc is involved in cell proliferation, death, differentiation, and the sensitivity of cancer cells to chemotherapy [26]. 10058-F4 inhibits c-Myc, regressing human acute myeloid leukemia, hepatocellular carcinoma, and ovarian cancer cells [9, 10, 27]. In pre-B acute lymphoblastic leukemia cells, 10058-F4 can also intensify the antileukemic effect of vincristine [11].

However, on account of its quick metabolism and low concentration within tumors, no substantial anticancer effect is observed in vivo following exposure of mice to either 20 or 30 mg/kg 10058-F4 [12]. Curcumin has been used to treat numerous types of cancer, including colorectal cancer, either alone or in conjunction with other treatments [28, 29], breast cancer [30, 31], lung cancer [32], prostate cancer [33], and liver cancer [34]. The potent antineoplastic properties of curcumin against different cancers are due to proapoptotic, antiproliferative, proapoptotic, and anti-inflammatory mechanisms [15, 16, 35]. Emerging preclinical research suggests that curcumin-based combination treatments improve anticancer activity without increasing toxicity. Banerjee et al. [36] observed that treating prostate cancer (PC3) (DU145 and PC3) cells with a combination of curcumin (20 mM) and docetaxel (10 mM) for 48 hours substantially decreased proliferation and promoted apoptosis in comparison to docetaxel and curcumin alone. A study based on HepG2 and PLC/PRF/5 cells found that a combination of curcumin (5 and 10 mM) and metformin (10 mM) can cause apoptosis and impede metastasis and invasion. Reduction of the epidermal growth factor receptor (EGFR)/STAT3 and NF–B/mTOR/Akt/PI3K inhibition of MMP2/9, vascular endothelial growth factor (VEGF), and vascular endothelial growth factor receptor 2 (VEGFR-2) and p53 and PTEN activation could all be contributors towards the anticancer effects.

Curcumin inhibits the expression of c-Myc in nonsmall cell lung cancer cells [36] and pancreatic cancer cells [24], in vitro and in vivo. In this work, we attempted to look into the impact of 10058-F4 combined with curcumin in PDAC, based on encouraging results obtained with c-Myc targeting techniques.

Consistent with previous reports [7, 8, 13], in most PDAC cell lines, c-Myc is amplified (Figure 1(a)). In vitro, 10058-F4 or curcumin alone reduced cell growth and induced apoptosis. Additionally, the combination-treated group's proliferation and apoptosis abilities were considerably altered (Figures 1(b) and 2). However, the 10058-F4 therapy had no discernible effect on the tumor burden. Compared to the control and 10058-F4 groups, combined curcumin plus 10058-F4 therapy substantially inhibited tumor growth (Figure 3). In the combination treatment group, the PCNA-positive cells were notably decreased, while the TUNEL-positive cells were considerably increased (Figure 4). This study also found that the combination of curcumin with 10058-F4 downregulated c-Myc and phosphorylation of Akt weakened Bcl-2 and Mcl-1 expression and increased Fas and cleaved-caspase 3 levels in SW1990 cells (Figure 5). Our findings show that curcumin induces tumor cell death and increases PDAC chemosensitivity to 10058-F4 through altering p-Akt and apoptosis-associated molecules. Importantly, our work furnishes sufficient in vivo evidence of the therapeutic potential of combined curcumin and 10058-F4 treatment in pancreatic cancer and shows cases a simple and convenient method for curcumin and 10058-F4 combinatorial therapy as a viable anticancer strategy in PDAC adjuvant therapy.

## 5. Conclusion

In conclusion, employing in vitro tests, we demonstrated the pharmacologic reduction of proliferation and induction of apoptotic effects of curcumin and 10058-F4, either alone or in combination. In vivo tests revealed that curcumin-induced tumor growth arrest boosted the anticancer efficacy of 10058-F4. However, additional tests, either in vivo or clinical trials, are a must to assess the effectiveness of the curcumin-10058-F4 combination and the safety of this technique in PDAC patients.

## Figures and Tables

**Figure 1:** c-Myc highly expressed in pancreatic cancer (a) examined the expression of c-Myc in 5 human pancreatic cancer cell lines (PANC-1, SW1990, BxPC3, Capan-1, and Capan-2 cells) and normal pancreatic epithelial cell hTERT-HPNE. (b) Cell viability was inhibited in the combination group.

**Figure 2:** Curcumin sensitized the anticancer influence of 10058-F4 in pancreatic cancer cells. (a) Colonogenic assay for the potent anticancer effect of combination. (b) Curcumin enhanced the sensitization the sensitization effect of 10058-F4 on SW1990 cells.

**Figure 3:** Tumor weight in the combination group and monotherapy groups.

**Figure 4:** Detection of cells in proliferation or apoptosis by PCNA and TUNEL staining.

**Figure 5:** Curcumin sensitized pancreatic cancer cells to 10058-F4 via inhibition of the Akt-modulated apoptosis pathway. (a) Protein levels of c-Myc and Akt phosphorylation in SW1990 cells treated with combination drugs and 10058-F4 alone. (b) Protein levels of Mcl-1 and Bcl-2 and the protein levels Fas and cleaved-caspase 3 in the combination treating group.

## Data Availability

The data used to support the findings of this study are available from the corresponding author upon request.
